The article "Study on Integration and Application of Artificial Intelligence and Wireless Network in Piano Music Teaching" was published in 2022. Journal: Comput Intell Neurosci.

# Study on Integration and Application of Artificial Intelligence and Wireless Network in Piano Music Teaching

**DOI:** 10.1155/2022/8745833

**Published:** 2022-05-14

**Authors:** Jiluo Li

**Affiliations:** School of Art, Zhengzhou Railway Vocational and Technical College, Zhengzhou 451460, Henan, China

## Abstract

Until 2019, most people had never faced the situation that would be their life-changing moment. Most universities are conducting classes for their students with the help of virtual classrooms indicating massive technological growth. However, this development does not take enough time to reach the students and the teaching person. Within five to six months of successful projects, most application producers have launched their official sites to conduct online classes and test ways for students. The introduction of virtual classes is not the only example of technological advancement; cloud computing, artificial intelligence, and deep learning have collaborated to produce appropriate, fine, and less error-prone results in all such fields of teaching. These technological advancements have given way to design models created with the wireless networks that are being made, particularly for music-related courses. The Quality-Learning (Q-Learning) Algorithm (QLA) is a pillar study for improving the implementation of artificial intelligence in music teaching in this research. The proposed algorithm aids in improving the accuracy of music, its frequency, and its wavelength when it passes. The proposed QLA is compared with the existing K-Nearest Neighbour (KNN) algorithm, and the results show that QLA has achieved 99.23% accuracy in intelligent piano music teaching through wireless network mode.

## 1. Introduction

A significant portion of China's educational system is devoted to the study of fine arts and crafts. Because of the introduction of artificial intelligence (AI) into the art school system, it is now required to make modifications to the piano curriculum [1]. Due to the high expense of piano lessons and the small number of students that enroll, piano instruction cannot be made more broadly available [2]. Online piano lessons have the potential to expand in popularity as a result of artificial intelligence and wireless networks, which is beneficial for the instrument as a whole [3]. By providing online piano instruction, artificial intelligence systems and network technology can increase the public's interest in piano art, as well as the art's societal influence.

Multiple linear regression and stepwise regression can be used to simplify the complex link between the difficulty of teaching and student achievement [4]. Explanatory approaches are also commonly used in research, which is not surprising. It appears that a student's ability to accomplish one particular feature may be associated with the difficulty of teaching that particular feature [5]. There has been little investigation into the categorical relationship between training complexity and feature performance. The association between difficulty in teaching and characteristic performance has been investigated by a number of researchers using a clustering technique that does not take into account the reference value of current barriers in the research process, as has been done by others [6]. There are a number of problems that must be overcome in order to compensate for human subjectivity in AI-guided piano instruction reform, including strengthening the elements that influence piano education and extracting them using an algorithm. The difficulty of instruction and the performance of pupils can both be quantified as a consequence of the use of a categorised technique.

The article "Study on Integration and Application of Artificial Intelligence and Wireless Network in Piano Music Teaching" was published in 2022. Journal: Comput Intell Neurosci.

For starters, a study may attempt to compensate for this challenge by failing to describe different variables adequately. This is supported by comparison studies and the Relief F weight approach, which are both based on the improvement of piano teaching-related characteristics and features [7]. Our research team has been successful in recognising all of the hierarchical influences of distinct piano instruction components through the application of metric learning theory and a new method known as KNN in Projected Feature Space (P-KNN). ML-SVM classification techniques and the Gaussian radial basis function (RBF) kernel method are utilised to find the parameters that affect piano training. Several other techniques, including logistic regression (LR), Lagrangian Support Vector Machine (LSVM), and Proximal Support Vector Machine (PSVM), are evaluated in relation to the P-KNN and ML-SVM algorithms, as well as PSVM [8]. It will take a significant amount of quantitative study to develop a piano teaching style that will have a specific reference value in the context of distance learning.

When artificial intelligence was first introduced to the music education field in the 1960s, new keyboard-based musical instruments were developed specifically for the purpose of teaching music. A wide range of musical styles can benefit from the timbres of the guitar, but rock & roll is undoubtedly the most well-known (mathematics, physics, etc.) [9]. These systems have many proponents, who are quick to stress how important it is to have professors who are motivated and worried about the consequences of granting credit to the wrong individuals. According to the majority of individuals, open-ended fields such as music production lend themselves well to logo design. However, there is no evidence to back up this allegation at this time. The Music Logo should be enhanced to accommodate a broader range of musical genres and composing approaches in addition to the current selection [10]. It is highly beneficial for intelligence tutoring systems to be aware of industry standards and goals, as well as strategies for identifying and classifying systemic problems. In terms of quality, there are just a handful of music venues that can compete with this. This has the potential to lead to the discovery of new musical domains with well-defined rules or objectives. In addition to audio training, it can be used in a variety of other applications. As long as the method's limitations are understood, it should never be used in an improper situation. Harmony Spaces is a human-centered technique that is based on artificial intelligence music ideas and methods [11]. The energy that powers this system comes from a multitude of sources. Harmony Space is more of a philosophy of music than a task paradigm for human-computer interaction, and it is based on that concept (harmony). The goal is to manipulate musical elements and relationships directly, with the domain theory being updated as needed to stay up with the most recent research findings [12]. It is possible to apply this strategy in a variety of scenarios. It would be exciting to see if the characteristics of group decision theory in other fields could be used to infer equal power for the interface as a research subject [13]. According to the researchers, MC cognitive assistance can be applied in a range of circumstances, including the creation of music [14]. A variety of factors contribute to the importance of harmony in our lives. It is possible to use the beautiful representations of harmony in Harmony Space to convey tonal and modal properties as well. These notions can be applied in a variety of musical contexts, as in the instance of MOTIVE, which is a rock band [15]. Due to the fact that it has an impact on a wide spectrum of corporate activities, bargaining is a popular issue for researchers in the fields of machine learning and artificial intelligence in educational settings. Students in the arts classroom can learn about the limitations of artificial intelligence concepts in music and do research on sentient cooperation [16]. Given the existing levels of domain expertise and visualisation abilities that are available to support human-machine connection, it is uncertain to what extent this work will be advantageous to music education under current delivery systems. Most of the time, students in music classes are forced to perform either a response to a question or a song that has been assigned by the teacher for them to reproduce [17]. The ability of students and teachers to collaborate more effectively is essential for a better musical experience. Students will be able to experience and understand music in ways that the teacher cannot because of the artificial intelligence system, rather than simply listening to the teacher's explanations [18]. Students of music can utilise this artificial intelligence application to learn about wireless communications and mobile computers, which is beneficial for their studies. In addition, students can gain an understanding of the fabrication process for the instruments [19]. When it comes to music training, both students and teachers can benefit from the use of artificial intelligence. A large number of innovative courses and teaching methods have been developed as a result of the introduction of intelligent instruments and software into music education programmes [20]. A growing number of music professors are instructing their students on how to play music, listen to music, and alter their own music. As a result, the quality of the students' work improves significantly [21]. It is possible to improve music education by better understanding the properties and behaviours of a network, such as musical symbols and elements. The advantages of online classroom learning are beneficial to both teachers and students in the field of music education [22]. Traditional musical conceptions are being called into question by the introduction of networked learning, which is transforming the way music is learned. Because of the advantages of the Internet, music education has spread throughout the world, culminating in the teaching of music education [23]. Because of the Internet, music teachers and students may now find additional resources for their classes. Because of the ease with which they can gather musical data and the speed with which they can do so, they are able to collect more and better data [24]. Therefore, students who learn by using the Internet may find themselves falling short of their educational objectives as a result of their use of the Internet. When learning music online, there are various advantages, including the availability of more music textbooks and the possibility for instructors to instruct students from a distance [25]. The researcher analyzed the strategies of piano teaching reform such as intelligent scoring, teaching, automatic playing function, and networked piano classroom [26]. The classification performance of multiclassification LSVM based on Gaussian RBF kernel is determined [27]. This study aimed at evaluating the integration of artificial intelligence with WSN in teaching piano music.

The article "Study on Integration and Application of Artificial Intelligence and Wireless Network in Piano Music Teaching" was published in 2022. Journal: Comput Intell Neurosci.

### 1.1. Motivation for the Study

We can see a tremendous development in the information technology sector in the recent technological era, which has caused all other sectors to work to face a revolution and profit. When compared to other organisations, educational departments have demonstrated the best use of technology in their teaching and learning processes. Music and musical instruments are difficult to teach and learn (TaL) for teachers and students in remote areas. The TaL of piano playing is studied in this study using the MIDI and Audio Edited for Synchronous TRacks and Organization (MAESTRO) Dataset. This dataset contains virtual recorded piano performances with notes labelled and audio waveforms. On the dataset, QL algorithm with artificial intelligence (AI) support is implemented to train the students. This algorithm is used on wireless networks (WN) to classify signal data after it has been recorded and updated. The algorithm combined with WN makes it easier for students to choose teachers.

## 2. Materials and Methods

Getting into the virtual music teaching concept, more than one technology is being involved in its growth, which is artificial intelligence, and this will not be considered the first time a different technology has been merged with music teaching. By 1960, AI was being used in music systems but not in the way of learning. It helps through discovering musical instruments with different sounds. Using the methods of deep neural networks, the music managing systems would look for such a pattern in the scoring pages. And here, bars are used to indicate the upcoming track. Once the artificial intelligence is merged with the music system, it will be able to create a separate set of mathematical rules. Involving the mathematical concepts is to create the original composition of the soundtrack. For example, consider the harmony spaces, which would relate the human interfacing modules to the artificial intelligence idea of music.

When the teaching methods are made online, it means the students or learners have a massive availability to access the notes given by the teaching personnel. If the classes are conducted in offline mode without any technology-based development in the class, then the students will not be able to go through their topics once they get out of the classes. In such a case, cloud storage makes the work more efficient for the students by allowing them to get back their testing and training work at any date and time. Normally, artificial intelligence is a kind of work in a separate world where, instead of human configuration, the technicians would create robots and assign tasks to the machines that benefit the humans who are living in the real world. Quality Learning is the AI algorithm that is one of the important concepts that stand behind music technology in all teaching fields. Creating an environment while at the same time making it understandable is mandatory. By increasing the cumulative reward with the help of the deep learning concept, the Q-learning algorithm plays a major role.

The article "Study on Integration and Application of Artificial Intelligence and Wireless Network in Piano Music Teaching" was published in 2022. Journal: Comput Intell Neurosci.

As a first step, teachers should be well versed in the teaching platform; only then will they be able to bring clarity to the student while delivering the concept. Even if the classes are made nonvirtual, it will be difficult for the students to grasp the concept if there is a lack of understanding with the teacher. According to the reaction, students would develop an interest in learning about the topic. Whatever the previous field has been shown in the learning platform, the Q-learning algorithm would bring massive growth to such a learning platform by increasing the efficiency and making analysis of the quality of music when it is delivered through wireless sensor networks. While hearing a tone on our mobile phones, the sound quality will differ when the same tone is being heard through an external speaker. So our prospect should be analyzing the frequency and serving it at the right time with actual bandwidth to the user who is located in a different location. With the help of Figure 1, the actual relations and the involvement of a student and the administrator will be analyzed. MAESTRO (MIDI and Audio Edited for Synchronous TRacks and Organization) is a dataset composed of about 200 hours of virtuosic piano performances captured with fine alignment (3 ms) between note labels and audio waveforms.

The creation of an intelligent piano playing instruction system based on wireless networks analyzes the piano education process's realisation technique. In addition, it offers a technique for measuring piano playing while employing a wireless network model for such issues in device piano teaching. That is, device teaching is a method of information transmission that does not involve communication. Furthermore, this document simulates the teacher's role in guiding students through the continuing playing method, which is essential in piano training.

Suppose there really are *u* training tests (*A*_*n*_,  *S*_*n*_) as particularly for identifying for the wireless sensor nodes, where *A*_*n*_ is the device's eigenvalue and *S*_*n*_ is the predicted data result. Assuming the aspect of the original signal is *t*, *A*_*n*_=(*n*_*n*1_, *n*_*n*2_,…, *n*_*nt*_) has been used to demonstrate its training examples of the *n* samples. *S*_*n*_=(*n*_*n*1_, *n*_*n*2_,…, *n*_*nt*_) is used to show the projected output sequence of the *n* sample. And *Q*_*n*_=(*Q*_*n*1_, *Q*_*n*2_,…,*Q*_*nt*_)^*S*^ is used to identify the *n* sample's evaluated output variable. The concentration between the *i* neurotransmitter and the adjacent *j* transmitter is *E*_*ij*_, where *j* is the lower limit of the *j* neuron.

The article "Study on Integration and Application of Artificial Intelligence and Wireless Network in Piano Music Teaching" was published in 2022. Journal: Comput Intell Neurosci.

When a transmitter is utilised as an inputs unit *Q*_*n*_=*A*_*n*_, the changes in the surface region WSN_*nj*_ of a *j* being transmitter can be defined as in equation

(1) $$\begin{array}{c} {\text{WSN}}_{nj}=\sum_{i}E_{ji}Q_{ni}-\theta_{j}, \end{array}$$

where *Q*_*ni*_ is the starting element's *i* transmitter output, *Q*_*ni*_ is the present element's *j* serotonin output, and *f*(WSN_*nj*_) is a Fourier transform. Equation (2) shows how to calculate *Q*_*ni*_.

(2) $$\begin{array}{c} Q_{ni}=\sum_{j=1}^{n}f\left({\text{WSN}}_{nj}\right). \end{array}$$

The development of these skills technique could also be utilised to train its *Q*_*ni*_ system using *D*_*n*_ as Sigmoid transfer function. The fundamental purpose of the training courses is to determine the nonlinear activation (refer to equation (3)).

(3) $$\begin{array}{c} D_{n}=\frac{1}{2}\sum_{j=1}^{r}{\left(l_{nj}-Q_{ni}\right)}^{2},\\ D=\sum_{n=1}^{u}D_{n}. \end{array}$$

Equation (4) is utilised in each training procedure Δ_*n*_, to lower the *E*_*ji*_ error value based on the gradient.

(4) $$\begin{array}{c} \Delta_{n}E_{ji}=\sum_{j=1}^{n}ŋ\delta_{nj}Q_{nj}+\sum_{j=1}^{r}{\left(l_{nj}-Q_{ni}\right)}^{2}. \end{array}$$

In equation (5), *ŋδ*_*nj*_ denotes the energy device.

(5) $$\begin{array}{c} \delta_{nj}=\sum_{j=1}^{r}{\left(l_{nj}-Q_{ni}\right)}^{2}-\sum_{j=1}^{n}\left(l_{nj}-Q_{nj}\right)Q_{nj}\left(1-Q_{nj}\right). \end{array}$$

Once *Q*_*nj*_ represents an activation functions unit, the calculation would be performed as shown in the following equation:

(6) $$\begin{array}{c} \delta_{nj}=\sum_{j=1}^{n}Q_{nj}\left(1-A_{nj}\right)\sum_{j}\delta_{nj}E_{ij}. \end{array}$$

Throughout sensor network teaching *h*_*nj*_, it is prudent to employ AI mean standard errors, as shown in the following equation:

(7) $$\begin{array}{c} AI=\frac{1}{tu}\sum_{t=1}^{u}\sum_{j=1}^{t}{\left({\hat{h}}_{nj}-h_{nj}\right)}^{2}. \end{array}$$

In equations (8) and (9), *n* denotes the value that connects the *j*^*th*^ hidden surface network to provide reduced weight matrices of a *β*_*j*_ hidden node and the inputs nodes.

(8) $$\begin{array}{c} Q_{nj}=\sum_{j=1}^{n}\beta h{\left(a+s+d\right)}^{1/2}, \end{array}$$

(9) $$\begin{array}{c} \sum_{j=r+1}^{n}\beta_{j}\left(g+a+A_{j}+d_{c}\right)=h_{i}. \end{array}$$

The rhythm sense is represented by *g* and *a* inside the dataset. The music frequency time is specified by *d*_*c*_.

The article "Study on Integration and Application of Artificial Intelligence and Wireless Network in Piano Music Teaching" was published in 2022. Journal: Comput Intell Neurosci.

The smart order is now on the lookout for a new area *A*_max_ − *A*_*i*_ inside its visual range. If the region *A* might be changed any further within the viewable region and also the normal satisfies *h*_1_ > *h*_2_ random behaviour may be evaluated using the following equation:

(10) $$\begin{array}{c} A_{j}=A_{j}+\text{random}\left(Vis\right)-if\left(h_{1}>h_{2}\right),A_{\text{inex}}=A_{i}+\text{random}\left(stp\right)*\left(A_{\max}-A_{i}\right). \end{array}$$

The random(*Vis*) specifies the visual range. It is comparable to the ∑_*q*=1_^*A*^*q*  *D*[*q*] intensity of a piano music audio. This is a measure of a music signal's tonality including its ∑_*q*=1_^*A*^*D*[*q*] spatial frequency elements. It is determined by using the following equation:

(11) $$\begin{array}{c} \text{Centroid}=\frac{\sum_{q=1}^{A}q\;D\left[q\right]}{\sum_{q=1}^{A}D\left[q\right]}. \end{array}$$

*D*[*q*] appears to be the amplitude. The following formula is used to compute the sequence-v spectral bandwidth by the following equation:

(12) $$\begin{array}{c} \text{Bandwidth}={\left(\sum_{q}Y\left(q\right){\left(f\left(q\right)-f_{d}\right)}^{v}\right)}^{1/v}. \end{array}$$

*Y*(*q*) denotes the spatial magnitude. It is the piano music level below ∑_*m*_signal[*b*(*o*)] − signal[*b*(*o* − 1)]*g*(*p* − *o*) where a significant portion of overall physical energy, 95%, can be discovered. It is calculated as in equations (13) and (14).

(13) $$\begin{array}{c} Ap=\frac{1}{2}\sum_{m}\text{signal}\left[b\left(o\right)\right]-\text{signal}\left[b\left(o-1\right)\right]g\left(p-o\right), \end{array}$$

(14) $$\begin{array}{c} \text{singnal}\left[b\left(p\right)\right]=\left\{\begin{array}{cc} 1, & P\left(p\right)\geq 0,\\ -1, & P\left(p\right)<0, \end{array}\right. \end{array}$$

and the direction is defined by *g*_*f*_, the input time is described by *b*_*f*_, the input vector just at a specified frequency was given by *b*_*t*_, and the outside situation is represented by *r*_*t*_. The piano music transistor information can be written in the following equation:

(15) $$\begin{array}{c} f_{t}=\sigma \left(g_{f}.\left[r.b_{t}\right]+b_{j}\right). \end{array}$$

*g* represents the matrix based on input entrance, and indeed *b*_*i*_ represents the neurotic period based on input entrance. Equation (16) represents the throughput entry.

(16) $$\begin{array}{c} \sigma_{t}=\sigma \left(g_{o}.\left[r_{t-1},b_{t}\right]+b_{0}\right). \end{array}$$

The heading corresponding to the an unknown point for piano music is denoted by *g*_*o*_, while the paranoid idea is denoted by *b*_*o*_. The following is the corresponding equation (17) presenting the calculation for the region $\tilde{d_{t}}$.

(17) $$\begin{array}{c} \tilde{d_{t}}=\tan\;r\left(g_{d}.\left[r_{t-1},b_{t}\right]+b_{c}\right). \end{array}$$

$\tilde{d_{t}}$ describes that current state of affairs on the inside. The WSN model's ultimate output targets are the piano music of a complex action of *o*_*t*_ and *d*_*t*_ which may be illustrated as in the following equation:

(18) $$\begin{array}{c} r_{t}=\sum_{t=1}^{d}o_{t}\tan\;r⊙\left(d_{t}\right). \end{array}$$

The article "Study on Integration and Application of Artificial Intelligence and Wireless Network in Piano Music Teaching" was published in 2022. Journal: Comput Intell Neurosci.

## 3. Results and Discussion

When a transmitter is utilised as an inputs unit *Q*_*n*_=*A*_*n*_, the changes in the surface region WSN_*nj*_ of a *j* as transmitter can be defined as in equation (1) based on this retrieved in Figure 2. It will be streamed of multiple signal classification for WSN algorithm with artificial intelligence in System Analysis, and there may be some signal latency.

The signal for recording audio in online mode is supposed to be a structural converter for students in this established framework. If a student detects any discrepancies in the audio, they can respond and critique it for future improvements. According to the text, AI will aid in the selection of different teachers and the playback of audio via the Wireless Sensor Network. The dataset's algorithms will be updated by AI. In result analysis on WSN with artificial intelligence, the proposed system has obtained standard score accuracy of 85% and command and interpret with overall accuracy of 89% in piano music memory along with overall accuracy of 93% (refer to Table 1).

*n* denotes the value that connects the *j*^*th*^ hidden surface network to provide reduced weight matrices of *β*_*j*_ hidden node and the inputs nodes as retrieved by Figure 3. The video is sent in audio but instead MIDI files, which have been coupled with 2(ms) testing the frequency into distinct musical pieces assembled including mean, standard error, and GB performance. CD-quality digital audio frequency for 45.1–47 kHz 18-bit PCM stereo is required. In the current technological era, there has been significant development in the information technology testing, which has prompted all other industries to work in order to face a revolution and profit. Educational departments have exhibited the test use of technology in their teaching and learning processes when compared to other organisations (refer to Table 2).

Prolog is a type that has a modelling process and the capacity to think intelligently. It is related to graphics with information technology understanding, and it includes propositions along with judgement comprehension scenarios. The phrase “Prolog programming” is commonly used in sets of data, ordinary mathematical results, completely credible, insufficient credibility, automatic recognition, and other fields. A new area *A*_max_ − *A*_*i*_ is inside its visual range. If the region *A* might be changed any further within the viewable region and also the normal satisfies *h*_1_ > *h*_2_ random behaviour may be evaluated using equation (10) retrieved from Figure 4 and Table 3. This is also widely used in music education and as a quantifier for mathematical expression vector for piano performance.

The article "Study on Integration and Application of Artificial Intelligence and Wireless Network in Piano Music Teaching" was published in 2022. Journal: Comput Intell Neurosci.

In this work, the organisers of the World Piano-e-Competition to create the raw data featured in this dataset are considered. Prolog operates on automatic representations throughout each competition installment, which is concert-reliable and credible pianos with just an array of high-quality MIDI capture and replay systems. The accuracy of the recorded MIDI data is strong enough that the competition's audition stage (see Table 3) can be judged remotely by hearing contestant performances replicated over the Internet on some other Prolog equipment.

Referring to Table 4 many of the overall evaluations of the audio signal are composed of piano music conveying communication signal characteristics (refer to Table 4). They are not qualitatively inspired and classify the distinctness of a rhythmic sensory signal in the sequence or frequency field. It is comparable to the ∑_*q*=1_^*A*^*q*  *D*[*q*] intensity of a piece of piano music. This is a measure of a music signal's tonality, including its ∑_*q*=1_^*A*^*D*[*q*] spatial frequency elements. It is determined by using equation (11) retrieved in Figure 5. Because music has such a wide range of variability biological feature extraction, associated musical frames are essential.

Audio wave signal's parameters are made up of several aspects of a piano music signal. They are not conceptually justified, nor do they classify the distinctness of a piano signal in the space-time or frequency field (see to Table 5). It is the piano music level below ∑_*m*_signal[*b*(*o*)] − signal[*b*(*o* − 1)]*g*(*p* − *o*) where a significance in Figure 6 portion of overall physical energy, 95%, can be discovered. Because music varies so much physiological feature extraction is done in brief intersecting skylights.

$\tilde{d_{t}}$ describes that current state of affairs on the inside. The WSN model's ultimate output targets are the piano music of a complex action, *o*_*t*_ and *d*_*t*_, which may be illustrated as retrieved in Figure 7. The steps for calculating an S3 score are as follows: Both of these performances are represented by reduced lettered components, whereas “Q” represents the query, or comparison, efficacy. Node (1) sorts performance results from equivalent to similar. Node (2) removes the most similar performances to leave an interference floor. Nodes (3) and (4) insert more comparable performance-related appearances one at a time to see how effectively they may obstruct the noise surface.

The article "Study on Integration and Application of Artificial Intelligence and Wireless Network in Piano Music Teaching" was published in 2022. Journal: Comput Intell Neurosci.

Incorporating stringed instrument recognition technology into children's piano studies can boost their interest in learning while also increasing the impact of piano education. Specifically, the model's performance for musical instrument recognition is improved in addition to developing the model on the basis of a neural network and refining its structure. The experimental results show that a multiple signal classification for WSN algorithm AI-based instrument identifying model may meet the criteria of piano teaching while also improving students' motivation in piano teaching. Reference to Table 6 provides the comparison of the existing KNN algorithm with the proposed Q-learning algorithm, and the results show that the proposed algorithm shows 99.23% of accuracy.

## 4. Conclusions

Recent technical advancements in the information technology sector have prompted all other industries to ramp up their efforts in preparation for revolution and profit. The educational sector has shown the best use of technology in its teaching and learning processes when compared to other organisations. Teachers and students in rural locations often have a tough time teaching and learning music and musical instruments. The MIDI and Audio Edited for Synchronous TRacks and Organization (MAESTRO) Dataset is used in this study to investigate piano playing's TaL. This set of data includes identified audio waveforms and virtual recordings of piano performances. Students are trained using Quality-Learning (QL) algorithm with AI help on the dataset. To identify signal data after it has been recorded and updated, this technique is employed on wireless networks (WN). The QL algorithm in conjunction with WN makes it easier for students to select their instructors. The study results proved that the proposed model outperforms better than the existing algorithms.

## Figures and Tables

**Figure 1:** Online teaching system as updated.

**Figure 2:** Performance of WSN with artificial intelligence in the System Analysis.

**Figure 3:** Performance analysis for frequency of use of Prolog language.

**Figure 4:** The multiple signal classification for WSN algorithm with artificial intelligence using analysis of frequency in affective dimension of music.

**Figure 5:** Performance analysis of teaching system's effect evaluation using multiple signal classification for WSN algorithm.

The article "Study on Integration and Application of Artificial Intelligence and Wireless Network in Piano Music Teaching" was published in 2022. Journal: Comput Intell Neurosci.

**Figure 6:** The piano music frequency analysis of teaching system's effect evaluation diagram.

**Figure 7:** Multiple signal classification for WSN algorithm performance analysis of piano music.

**Table 1:** Result Analysis WSN with artificial intelligence in the System Analysis.

Parameter	Multiple signal classification for WSN algorithm	Structure converter	Database	Accuracy (%)
Standard score	178	255	463	85
Command and interpret	184	278	455	89
Music memory	197	247	574	93

**Table 2:** Result analysis for frequency of use of Prolog language.

	Mean	Standard deviation	Size (GB)
Testing	2.54	375	75.83
Frequency	2.67	262	49.42
Database	2.14	342	58.67

**Table 3:** Performance analysis of frequency of use of Prolog language.

	Language in Prolog	Automatic representation	Mathematical result
Suggestion	1443	278	114
Experienced professional	1316	249	125
Dataset	1502	236	147
Ordinary reliable	2315	236	161
Inadequate credibility	2539	423	145
Totally credible	1556	262	153

**Table 4:** Overall evaluation and test piano teaching system and experimental results.

Piano teacher	Overall evaluation	Communication command	Rhythm sense
Music 1	0.956	0.723	0.856
Music 2	0.823	0.835	0.821
Music 3	0.971	0.878	0.842
Music 4	0.974	0.989	0.979
Music 5	0.949	0.848	0.845
Music 6	0.947	0.846	0.756
Music 7	0.889	0.873	0.734
Music 8	0.824	0.789	0.876
Music 9	0.712	0.843	0.951
Music 10	0.943	0.9	0.87

**Table 5:** Frequency analysis for piano music teaching education.

Piano teacher	Time (s)	Frequency	Rhythm sensation
Music 1	0.657	0.663	0.712
Music 2	0.712	0.576	0.743
Music 3	0.783	0.652	0.618
Music 4	0.764	0.721	0.565
Music 5	0.699	0.678	0.687
Music 6	0.665	0.698	0.634
Music 7	0.743	0.612	0.673
Music 8	0.716	0.767	0.667
Music 9	0.715	0.649	0.795
Music 10	0.823	0.599	0.691

**Table 6:** Comparison result analysis for existing system.

Algorithm	Time (s)	Frequency in rhythm sensation	Training/testing (%)	Overall accuracy (%)
Q-learning algorithm	1.5	0.912	0.599	99.23
Existing method: KNN	4.1	0.967	0.678	94.46

## Data Availability

The data used to support the ﬁndings of this study are available from the corresponding author upon request.
